The article "SRSF3 Restriction Eases Cervical Cancer Cell Viability and Metastasis via Adjusting PI3K/AKT/mTOR Signaling Pathway" was published in 2022. Journal: Contrast Media Mol Imaging.

# SRSF3 Restriction Eases Cervical Cancer Cell Viability and Metastasis via Adjusting PI3K/AKT/mTOR Signaling Pathway

**DOI:** 10.1155/2022/8497078

**Published:** 2022-09-26

**Authors:** Lirong Zhang, Jing Li, Liping Zhang

**Affiliations:** Department of Gynecology, Wuhan Childrens Hospital, Wuhan Maternal and Child Health Hospital, Wuhan Womens and Childrens Health Care Center, Wuhan, Hubei Province, China

## Abstract

**Objective:**

To investigate the effect of SRSF3 on the viability and metastasis of cervical cancer (CC) SiHa and Hela cells.

**Methods:**

In vitro, HeLa cells and SiHa cells were cultured. In cervical cancer cells, RNA interference technology was utilized to lessen the SRSF3 level, and via RT-PCR utilization, the SRSF3 level in every group of cells was revealed. By employing the CCK-8 method, the OD value was revealed in every group at 24, 48, 72, and 96 h. On the migration of cervical cancer SiHa and HeLa cells via transwell utilizing, the consequence of SRSF3 was surveyed. Through western blotting utilizing, the PI3K/AKT/mTOR signaling pathway-connected proteins levels was revealed.

**Results:**

In SiHa cells, contrasted to the NC-SiHa group, the SRSF3 level, the number of invasive cells per unit area, the p-PI3K/PI3K level, the p-AKT/AKT level, and the p-mTOR/mTOR level in the si-SRSF3 group were substantially lessened. The OD value at 490 nm of the si-SRSF3 group had no impressive divergence, contrasted to the NC-SiHa group at 24 h. At 48 h, the OD value of the si-SRSF3 group was impressively lessened than that of the NC-SiHa group. This connection was time-dependent. In HeLa cells, the SRSF3 level, the number of invasive cells per unit area, the level of p-PI3K/PI3K, the level of p-AKT/AKT, and the level of p-mTOR/mTOR in the cells of the si-SRSF3 group in the NC-HeLa group were impressively lessened than those in the NC-Hela group. Between the NC-HeLa group and the si-SRSF3 group at 24 h, there was no impressive divergence in the OD value at 490 nm. At 48 h, the OD value of the si-SRSF3 group was impressively lessened than that of the NC-SiHa group. This connection is time-dependent.

**Conclusion:**

Reducing the SRSF3 level can restrain the viability and metastasis of cervical cancer cells via restraining the PI3K/AKT/mTOR signaling pathway.

## 1. Background

Cervical cancer (CC) is one of the most common malignant tumors of the female reproductive system, with the second highest incidence rate among female malignancies, just below breast cancer [1]. Owing to the current situation of multiple sexual partners, early sexual intercourse, and the increase of carriers of the high-risk human papillomavirus, the quantity of female CC sufferers in China is increasing year after year and disclosing a trend of gradual rejuvenation [2]. Many genes are aberrantly expressed in CC sufferers, such as P53, STIL and SRSF3, also known as serine and arginine-enriched splicing factor 3, a member of the RNA-binding protein family and the smallest protein in the highly conserved SR family [3]. SRSF3 has the ability to actively splice with many mRNAs while at the same time enabling the splicing of its own mRNAs to lessen its own protein level [4]. Lu et al. [5] have disclosed that SRSF3 has a connection with the cell cycle and apoptosis and that reducing the SRSF3 level restrains cell growth, arrests the cell cycle in the G2/M phase and boosts apoptosis. Current studies have disclosed that SRSF3 is closely connected with the progression and progression of many tumors, usually disclosing high levels in ovarian cancer, CC, and colon tumor tissues [6, 7]. Based on this, we hypothesized that reducing the SRSF3 level in CC cells might restrain their viability and boost their apoptosis. Therefore, we utilized siRNA technology to interfere with the SRSF3 level in CC cells, to reveal its viability and metastatic ability, and to reveal its connected pathways to survey the consequence of SRSF3 restriction on CC and its mechanism of action, so as to supply strong evidence for SRSF3 restriction in CC cells.

The article "SRSF3 Restriction Eases Cervical Cancer Cell Viability and Metastasis via Adjusting PI3K/AKT/mTOR Signaling Pathway" was published in 2022. Journal: Contrast Media Mol Imaging.

## 2. Methods

### 2.1. Cell Recovery and Culture

The SiHa cells and Hela cells (Shanghai Cell Bank of the Chinese Academy of Sciences) that were stored in liquid nitrogen were taken out and quickly thawed in a constant temperature water bath at 37°C. 1 mL of 89% RPMI 1640 (Guangzhou Weijia Technology Co., Ltd), 10% fetal bovine serum and 1% of 100 U/mL penicillin-streptomycin were mixed and augmented to 5 mL of bacteria-free EP. Cells were diverted to an EP in an ultraclean table, gathered via centrifugation at 1000 r/min with 3 min, at 37°C, rinsed twice with sterile PBS prewarmed, resuspended with complete medium and diverted to a culture dish, and incubated in a cell culture incubator at 37°C and 5% CO_2_. The following day the medium was replaced with a new complete medium, dead cells and cell debris were taken out, and the washed cells were continued in culture, digested with 0.25% trypsin when the cell density exceeded 75% and passaged at a ratio of 1 : 3.

### 2.2. Cell Transfection

SiHa and Hela cells were inoculated in 6-well plates at a density of 5 × 10^5^ cells/well and cultured after transfection of control RNA and 10 nmol/siRNA (Santa Cruz Corporation, USA) into the cells employing Lipofectamine 2000 (Invitrogen), respectively. After 48 h, the cells were passaged and transfected again, and the protein levels of every group of cells were measured after 96 h.

The article "SRSF3 Restriction Eases Cervical Cancer Cell Viability and Metastasis via Adjusting PI3K/AKT/mTOR Signaling Pathway" was published in 2022. Journal: Contrast Media Mol Imaging.

### 2.3. Gene Level Detection via RT-PCR

SiHa cells and Hela cells were gathered in culture up to log phase, counted, cell density was adjusted, and cells were inoculated in 6-well plates at a density of 5 × 10^5^ cells/well. When the cells had revealed about 50% growth, the medium was changed, and the cells were grouped and treated for drug administration. After 48 h of drug treatment, cell samples were gathered, and RNA was extracted from the cell samples according to the steps of the RNA extraction kit. After revealing the concentration, reverse transcription was conducted, and cDNA samples were obtained. Finally, SRSF3 levels were revealed according to the qPCR instruction steps, employing *β*-actin as an internal reference control (Table 1).

### 2.4. CCK-8 Detection of Cell Viability

SiHa cells and Hela cells were gathered at the log phase. After 24 hours of adherent culture, 10 *μ L* CCK-8 solution was added to each well. The cells were incubated for 2 h in a suitable in vitro environment, and the viability of the cells was ascertained via the OD value at 490 nm employing an enzyme marker.

### 2.5. Transwell Assay for Cell Metastasis

SiHa and Hela cells were cultured to logarithmic phase, and the cell density was adjusted to 5 × 10^5^ cells/mL. The upper layer of the chambers was cultured in RPMI 1640 medium, and the lower layer of the chambers was augmented to a normal culture medium. After 24 h of incubation, from the vesicles with sterile cotton swabs, cells were taken out, and cells that had invaded the lower layer of the vesicles were stained with crystal violet, and five fields of view per well were randomly picked for counting. 3 replicate wells per group, experiment repeated at least 3 times.

### 2.6. Western Blotting to Reveal Relevant Protein Level

SiHa and Hela cells were cultured to log phase and adjusted to a cell density of 5 × 10^5^ cells/mL and inoculated in 6-well plates. Via the protein extraction kit procedure, total protein was extracted from the cell samples, and the total protein concentration was ascertained via the BCA protein quantification method. Mixed with the loading buffer, and then conducted SDS-PAGE for 10 min at 95°C in a metal bath (80 V, 40 min, 120 V, 50 min); membrane metastasis (metastasis of proteins to PVDF membrane via electro metastasis); closure (incubation at room temperature for 2 h with 5% skimmed milk powder); 1 × TBST for membrane rinsing. Augmented PI3K, p-PI3K, Akt, p-Akt, m TOR, p-mTOR and *β*-actin antibodies (dilution ratio 1 : 1000, Abcam) and incubated for 8 h at 4°C; rinsed the membrane. The secondary antibody (dilution ratio 1 : 2000, Abcam) was augmented and incubated at 37°C for 2 h. ECL chemiluminescence reagent (Bio-Rad, USA) was utilized for colour progression, and *β*-actin was utilized as an internal reference control to reveal protein level.

The article "SRSF3 Restriction Eases Cervical Cancer Cell Viability and Metastasis via Adjusting PI3K/AKT/mTOR Signaling Pathway" was published in 2022. Journal: Contrast Media Mol Imaging.

### 2.7. Statistical Methods

The software utilized for data analysis and graphing in this study was SPSS 22.0 and GraphPad Prism 8.0, and ANOVA was conducted employing one-way ANOVA, with *P* < 0.05 implying statistically impressive divergences.

## 3. Results

### 3.1. Level of SRSF3 in All Groups of Cells

RT-PCR was utilized to reveal the SRSF3 level in every group of cells, and it was found that in SiHa cells, as contrasted to the NC-SiHa group, the SRSF3 level was impressively lessened in the si-SRSF3 group of cells (*P* < 0.01). In HeLa cells, contrasted to the NC-SiHa group, SRSF3 level was impressively lessened in the si-SRSF3 group of cells (*P* < 0.01), Figure 1.

### 3.2. Cell Viability in Every Group

CCK-8 assay of OD values for every group of cells revealed that in SiHa cells, in the si-SRSF3 group, the OD value at 490 nm was impressively lessened than that in the NC-SiHa group at 24 h (*P* < 0.05). In the si-SRSF3 group, the OD value at 490 nm was impressively lessened than that in the SiHa group after 48 h (*P* < 0.01). In HeLa cells, in the si-SRSF3 group, the OD at 490 nm was impressively lessened than that in the NC-HeLa group at 24 h (*P* < 0.05). After 48 h, in the si-SRSF3 group, the OD value at 490 nm was impressively lessened than that in the NC-HeLa group (*P* < 0.01), Figure 2.

### 3.3. Migration of Cells in Every Group

Transwell assay was utilized to reveal the numberof cells per unit area of invasion in every group. In SiHa cells, contrasted to the NC-SiHa group, the numberof cells per unit area of invasion was impressively lessened in the si-SRSF3 group (*P* < 0.01). In HeLa cells, contrasted to the NC-HeLa group, the numberof cells per unit area that underwent invasion was impressively lessened in the si-SRSF3 group (*P* < 0.01), Figure 3.

### 3.4. PI3K/AKT/mTOR Signaling Pathway Profile

In all groups of cells, a western blotting assay was utilized to reveal PI3K/AKT/mTOR signaling pathway-connected proteins levels. Contrasted to the NC-SiHa group, in SiHa cells, p-PI3K/PI3K levels, p-AKT/AKT levels, and p-mTOR/mTOR levels were impressively lessened in the si-SRSF3 group (*P* < 0.01). In HeLa cells, contrasted to the NC-HeLa group, p-PI3K/PI3K levels, p-AKT/AKT levels, and p-mTOR/mTOR levels were impressively lessened in the si-SRSF3 group (*P* < 0.01); see Figure 4.

## 4. Discussion

CC is a common and highly prevalent malignant tumor of the female reproductive system that seriously influences women's wellness and worth of living [8]. In novel years, as research has progressed, there have been more breakthroughs regarding CC, but the biological characteristics of the cells influencing CC have not yet been fully characterised in terms of their mechanism of action. CC has a strong proliferative and invasive capacity, which is an important reason why sufferers are difficult to treat and have a poor prognosis. The main routes of metastasis in CC include direct metastasis, hematogenous metastasis and lymphatic metastasis [9, 10]. Therefore, exploring the biological characteristics of the cells of CC is a current research hotspot. Deng et al. [11] have disclosed that there is aberrant variable splicing in the typical biological processes of tumors and that this aberrant variable splicing is closely connected to processes such as tumor viability and apoptotic escape. SRSF3 can conduct self-splicing as well as active splicing of a wide range of genes, and currently, common spliceable genes include SRSF5, ILF3, and HER2 [12]. It has now been disclosed that SRSF3 is highly expressed in CC. Based on this, we hypothesized that reducing the SRSF3 level in CC cells could modulate the malignant biological features of CC. In this study, two different CC cells were picked: SiHa cells and HeLa cells, and the gene interference technique was utilized to lessen the SRSF3 level in these two cells to reveal the malignant biology of these two cells and to investigate the section of SRSF3 in CC cells.

The article "SRSF3 Restriction Eases Cervical Cancer Cell Viability and Metastasis via Adjusting PI3K/AKT/mTOR Signaling Pathway" was published in 2022. Journal: Contrast Media Mol Imaging.

In this study, after employing interfering RNA to lessen the SRSF3 level in SiHa cells and HeLa cells, PCR was utilized to reveal the SRSF3 level in every group of cells, and the SRSF3 level in both cells was impressively lessened after employing interfering RNA, implying the success of the interfering RNA technique utilized in this study. Lin et al. [13] have disclosed that SRSF3 is capable of splicing MAP4K4 in colorectal cancer cells and is an important proto-oncogene with a regulatory section in cell viability and cycle. Therefore, in this study, the CCK-8 assay was utilized to reveal cell viability in every group of cells. In the experiment, the OD of the cytosol was measured via an enzyme marker. A higher OD value implies more microorganisms implying a more viable cell. In this study, the activity of the two CC cells transfected with the blank plasmid and the cells transfected with the interfering plasmid did not differ impressively within 24 h after transfection. After 48 h, it could be found that the OD value of the cells in the si-SRSF3 group transfected with interfering SRSF3 level was impressively lessened than that of the cells in the group transfected with the blank plasmid, and the OD value of the cells in the group transfected with the interfering plasmid continued to decrease impressively with time. It implies that reducing the SRSF3 level can effectively restrain the viability of CC cells. This may be related to the fact that SRSF3 can improve SPAG5 level, and lessening SRSF3 level leads to a notable SPAG5 decrease in CC cells; SPAG5 is an important factor arranged on the equatorial plate to restrain spindle disorder and multi-polarization. The decrease in SPAG5 level will make the chromosomes of cells unable to normally arrange on the equatorial plate during mitosis and make cell division blocked in the G2/M phase, which will restrain the viability of tumor cells and lessen cell activity.

The article "SRSF3 Restriction Eases Cervical Cancer Cell Viability and Metastasis via Adjusting PI3K/AKT/mTOR Signaling Pathway" was published in 2022. Journal: Contrast Media Mol Imaging.

The malignant biological characteristics of tumors include metastasis in addition to malignant viability [14]. Based on this, the Transwell cell experiment was utilized to reveal the metastatic ability of cells in every group. Contrasted to the transfected blank cell group, the number of cells invaded per unit area in the si-SRSF3 group was impressively lessened, which disclosed that reducing the SRSF3 level could effectively lessen the metastatic ability of tumors. This may be because SRSF3 has the function of shearing vascular endothelial growth factor and produces two isomers. There is an antiangiogenesis consequence in these two isomers, which restrains the mesenchymal transformation of tumor cells and limits the metastatic ability of tumor cells. Che and Fu [15] have disclosed that SRSF3 plays a section in promoting cell viability in tumor cells, with higher levels in tumor cells with a high degree of malignancy, and the conclusions revealed in this study are similar to theirs.

This study further investigated the molecular mechanisms underlying the consequences of SRSF3 on the malignant biological characteristics of CC tumor cells. Studies have disclosed that PI3K/AKT/mTOR signaling pathway is involved in the viability, differentiation, apoptosis, aging, and other processes of a variety of tumor cells [16, 17]. mTOR is the target molecule of rapamycin, the confluence point of the upstream autophagy pathway, and the main regulatorysignal of autophagy. When it is phosphorylated, it forms Atg13, which makes it unable to combine with Atg1 to form autophagosome, boosts the adhesion of ribosomes to the endoplasmic reticulum, and restrains the fall off of the endoplasmic reticulum membrane to form autophagosome membrane [18]. PI3K/Akt is one of the upstream pathways regulating mTOR. The upstream PI3K can effectively block the downstream Akt and mTOR, and Akt can be activated via PI3K and mTOR directly [19]. When the upstream PI3K is restrained, the downstream Akt and mTOR will be restrained, which will make the endoplasmic reticulum membrane of CC cells fall off, thus promoting cell apoptosis. In this study, PI3K/AKT/mTOR signal pathway connected proteins levels were revealed. It was found that p-PI3K/PI3K level, p-AKT/AKT level and p-mTOR/mTOR level were impressively lessened in the si-SRSF3 group, implying that PI3K phosphorylation was restrained, resulting in the restriction of Akt and mTOR. It discloses that restraining the SRSF3 level can restrain the PI3K/AKT/mTOR signaling pathway, thereby regulating the biological characteristics of CC cells. Wang et al. [20] have disclosed that the viability, apoptosis, and invasion of cervical cancer cells can be influenced via restraining PI3K/AKT/mTOR signal pathway, and the conclusion of this study is similar to it.

The article "SRSF3 Restriction Eases Cervical Cancer Cell Viability and Metastasis via Adjusting PI3K/AKT/mTOR Signaling Pathway" was published in 2022. Journal: Contrast Media Mol Imaging.

To sum up, reducing the SRSF3 level in CC cells can effectively restrain its viability and lessen its metastatic ability. Its mechanism may be connected to the restriction of the PI3K/AKT/mTOR signal pathway, but this study has not yet involved the PI3K/AKT/mTOR connected pathway. Later, we will continue to survey other connected signal pathways involved in SRSF3 and further supply strong evidence for SRSF3 to restrain CC cells.

## Figures and Tables

**Figure 1:** Level of SRSF3 in every group of cells. Contrasted to the NC group ^*∗∗*^*P* < 0.01.

**Figure 2:** Cell viability in every group. Contrasted to the NC group ^*∗*^*P* < 0.05; Contrasted to NC group ^*∗∗*^*P* <  0.01.

**Figure 3:** Migration of cells in every group. Contrasted to the NC group ^*∗∗*^*P* < 0.01.

**Figure 4:** PI3K/AKT/mTOR signaling pathway profile. Contrasted to NC group ^*∗∗*^*P* < 0.01.

**Table 1:** Primer sequences.

Grouping	Upstream primer	Downstream primer

SRSF3	5′-CCCTCGAGGGAAGACCAGTTTGCAAGAGGAGTGGT-3′	5′-ATTTGCGGCCGCTTTATAGCTGGGCAGGAGTTAAGAGG-3′
*β*-actin	5′-CACCATTGGCAATGAGCGGTTC-3′	5′-AGGTCTTTGCGGATGTCCACGT-3′

## Data Availability

The datasets used and analyzed during the current study are available from the corresponding author upon reasonable request.
